The article "Assembly of 97 Novel Bacterial Genomes in the Microbial Community Affiliated with Polyvinyl Alcohol in Soil of Northern China" was retracted in 2024. Reasons: suspected computer-generated content; unreliable results or conclusions; concerns about the data; concerns about the results or conclusions.

# Assembly of 97 Novel Bacterial Genomes in the Microbial Community Affiliated with Polyvinyl Alcohol in Soil of Northern China

**DOI:** 10.1155/2022/2229147

**Published:** 2022-01-18

**Authors:** Jiaxing Liu, Xun Gu, Hui Li

**Affiliations:** ^1^MOE Key Laboratory of Contemporary Anthropology, School of Life Sciences, Fudan University, Shanghai 200438, China; ^2^Department of GDC Biology, Iowa State University, Ames, IA 50014, USA

## Abstract

**Background:**

Undeveloped ecosystems belong to rich source of microbial population, of which resources remain unearthed. A kind of polymeric compound system with high polyvinyl alcohol (PVA) content has been reported and named *Taisui*. Marker gene amplification showed that *Taisui* harbored little-explored microbial communities.

**Aim:**

To address this issue, our study attempted to recover draft genomes and functional potential from microbial communities in *Taisui* using the metagenomic approach. *Material and Methods*. *Taisui* communities provided 97 novel bacterial genomes from 13 bacterial phyla, including bacteria candidate phylum. Two novel genus-level lineages were recovered from Planctomycetes and Chloroflexi. Based on the draft genomes, we expanded the number of taxa with potential productions of PKS and NRPS in phyla including Candidatus Dadabacteria, Chloroflexi, and Planctomycetes.

**Results:**

A rich diversity of PVA dehydrogenase genes from 4 phyla, involving Proteobacteria, Acidobacteria, Acitinobacteria, and Planctomycetes, were identified. The phylogenetic tree of PVA dehydrogenase showed the possibility of horizontal gene transfer between microbes.

**Conclusion:**

Our study underscores the substantial microbial diversity and PVA degradation potential in the previously unexplored *Taisui* system.

## 1. Introduction

Polyvinyl alcohol (PVA) is a common water-soluble polymer for farming, packing, fiber coating, etc. Due to the high mass of production and utilization, PVA pollution in the environment was considerable, especially in the major production regions: China, the USA, Western Europe, and Japan [1, 2]. For PVA degradation with less cost and sludge generation, bacterial PVA-degraders were isolated from PVA-containing systems [2]. However, symbiotic behaviors of PVA degrading microbes make the study of microbial community in PVA-containing systems be needed. A kind of underground polymeric compound (named “*Taisui*”) system has been reported recently [3]. Chemical analysis showed that this system can be characterized by high level of PVA or a mixture of PVA and polyacrylic acid [3]. The distribution of *Taisui* has been analysed through finding reports from 1992 to 2015. More than 60% of *Taisuis* existed in soil layers, and more than 60% of them were in northern China [4].

The PVA-containing system of *Taisui* can be a valuable object of metagenomic analysis. First, *Taisui* has stable morphological characteristics and internal structures [3]. Like a bioreactor, the structure of *Taisui* (Figure S1) separates microbial populations from surrounding environments. Second, *Taisui* has stable chemical compositions [3], which indicates stable microbial pattern. Third, *Taisui* systems harboring little-explored microbial communities. Previous research has shown that *Taisui* hosts a rich diversity of novel microbes [3]. More than 40% bacterial OTUs in 2 samples were unclassified at the phylum level, and more than 75% fungal OTUs in 8 samples were unclassified. Metagenomic sequencing can bypass the cultivation bottleneck by obtaining metagenome-assembled genomes (MAGs), leading to the discovery of novel microbial diversity and new metabolisms from challenging systems [5, 6]. Based on these prior observations, we inferred that *Taisui* systems offered an opportunity for expand microbial diversity and PVA biodegradation. In this study, we reconstructed MAGs from metagenome of *Taisui* samples and investigated PVA degradation potential of *Taisui* microbiota. The results show the wealth of evolutionary diversity in unexplored systems, markedly expand the diversity of PVA dehydrogenase, and will contribute to future comparative studies of PVA polluted environments.

## 2. Material and Methods

### 2.1. Sample Collection

Four *Taisui* samples included in this study were collected from Jinzhou (Liaoning province), Baotou (Inner Mongolia), and Aksu (Xinjiang Province, Figure 1(a)). The *Taisui* individuals were washed using fresh water after being dug out from the soil layer, and the entire of them were delivered at room temperature (about 15°C). For each *Taisui* individual, four samples were collected in the meantime. The samples were collected both from the outside (the surface of *Taisui*) and the inside (about 5 cm depth from the outside) in equal quantity (2∗2∗2 cm of each). The samples, belonging to one *Taisui* individual, were pooled as one sample for future investigation. To observe the structure of *Taisui*, the TS.JZ1 sample was used as a representative sample for microscopic observations. Photographs were taken using a digital camera mounted on a light microscope.

### 2.2. DNA Extraction and Sequencing

Before DNA extraction, we used 1% dimethyl sulphoxide and dry bath to remove polyvinyl alcohol. DNA extraction referred to the phenol-chloroform extraction [7] was described in the supplement. After DNA purification, equal volumes of isopropanol at +4°C (100%) were added to the upper phase previously transferred into a clean 1.5 ml tube, then tubes were slowly mixed by inversion and kept overnight at -20°C, before another centrifugation (15 min at 16000 × g). Following removal of the supernatant, 1 ml of 70% ethanol at +4°C was added to the DNA pellets. These pellets were suspended by flicking the tubes, followed by inversion and centrifugation (15 min at 16000 × g), then pellets were dried for 10 min (V-AQ mode, Vacufuge plus, Eppendorf), and 50 *μ*l of nuclease-free water was added. Samples were shotgun-sequenced for metagenomics on the Illumina HiSeq platform at Novogene (Tianjin, China), and paired-end reads were generated. For HiSeq sequencing, each sample can be barcoded (added during library preparation), and equal quantities of barcoded libraries can be multiplexed during sequencing. HiSeq reads are aligned to a cohort of nonredundant National Center for Biotechnology Information (NCBI) complete genomes using the Short Oligonucleotide Analysis Package (SOAP) alignment tool29, which is typically faster to run than the Basic Local Alignment Search Tool (BLAST) or the BLAST-like Alignment Tool (BLAT). Genome coverage is calculated using the SOAP.coverage package.

### 2.3. De Novo Assembly and Analysis

The quality control of the metagenomic reads was performed using FastQC [8] and MultiQC [9]. Adapters and low-quality reads were removed. We set the minimum base quality score of 38. Bases with quality score < 38 were treated as low-quality bases. Reads were filtered as long as they contained more than 40 bp of low-quality bases. We also removed reads that contained more than 10 bp of N and reads that overlapped more than 15 bp with adapters to generate clean data. The high-quality reads were de novo assembled into contigs by using MEGAHIT [10] with default settings. We used QUAST [11] to evaluate metagenomic assemblies.

Assembled contigs were used to predict open reading frames (ORFs) using Prokka [12] with annotation mode included archaea, bacteria, mitochondria, and viruses. To get the nonredundant ORF dataset, the ORFs of four samples were merged, and the redundant ORFs were removed using CD-HIT [13, 14]. The abundance of ORFs in each sample was calculated using Salmon [15]. The ORFs were taxonomically annotated against the NCBI GenBank nonredundant protein sequence (nr) database using DIAMOND (*E*-value 1e-5) [16]. Taxonomic annotations were generated using MEGAN6 [17], with the maximum e-value cutoff as 1e-5. For KEGG and COG annotation, the ORFs were searched against eggNOG database using eggNOG-mapper [18]. Besides, the ORFs that encode carbohydrate-active enzyme (CAZyme) domain were profiled by mapping against CAZy database [19] using DIAMOND (*E*-value 1e-5).

Shannon-Weaver index, Simpson's index, Shannon evenness index, and Bray-Curtis index of all taxa at the species level were estimated using Vegan. UPGMA clustering of samples was obtained using SplitsTree4 [20]. The clustering tree and bar plots were edited in iTOL [21].

### 2.4. Meta-Pathway Reconstruction

The meta-pathways were the combination of metabolic pathways of multiple bacteria in the metagenomic dataset. The meta-pathways were reconstructed based on the functional annotation of ORFs (generated using eggNOG database and CAZy database). Also, the KEGG pathways were profiled using Pathview [22] for reconstruction. To evaluate the contribution of bacteria to a given enzyme in the metabolic pathways, the taxonomic annotation of ORFs (generated using NCBI-NR database) was combined with the functional annotation.

### 2.5. Metagenomic-Assembled Genome

Coassemblies were binned using MetaWRAP (parameters: -c 70 -x 5) [23], which called concoct, maxbin2, and metabat2 for binning at the same time. Bin refinement was performed based on the results of these binning software packages using “bin_refinement.” Reads were aligned to contigs using BWA to generate separate files for each cluster. Separated reads were then reassembled using “reassemble_bins,” and final beat bins were obtained based on the results of CheckM [24], which resulted in a final set of 97 bins.

Using CheckM, bins were filtered for completeness ≥70% and contamination ≤5%. Taxonomy was assigned to genome bins using GTDB-Tk [25]. The amino acid identity (AAI) between MAGs was calculated by CompareM v. 0.1.1 [26]. The replication of MAGs was checked at 95% average nucleotide identity (ANI) to generate the species number using pyani [27, 28]. According to the standards suggested by Glendinning et al. [29], genomes were defined as novel strains (GTDB-Tk ANI output < 99%), novel species (GTDB-Tk ANI output < 95%), and novel genera (all MAGs clustered at 60% AAI [30] without a genus GTDB-Tk assignment).

For MAG phylogenetic analysis, the concatenated sequence alignment of core marker genes was built by Up-to-date Bacterial Core Gene pipeline (UBCG) [31]. Conserved blocks were selected from multiple alignments by Gblocks (parameters: -b5 h) [32] for further analysis. The best-fit evolutionary model was selected using ModelTest-NG [33]. The phylogenetic tree was inferred using RAxML-NG [34] with the GTR + I + G4 model. Node support was generated through 500 bootstrap replicates. The phylogenetic tree was finalized for publication using iTOL website [21].

For the phylogenetic placement analysis, the MAGs and reference genomes from NCBI database belonging to the phyla Planctomycetes and Chloroflexi were selected. To build the tree of Chloroflexi, we selected 15 genomes involving complete genomes of Anaerolineae, Ardenticatenia, and Dehalococcoidia (part of Dehalococcoidia complete genomes were selected according to the results of GTDB-Tk), and closely related genome (UBA2991) of MAGs according to GTDB-Tk. And for the tree of Planctomycetes, we selected 48 genomes involving complete genomes of Planctomycetia, Phycisphaerales, and genomes of UBA1135, UBA1845, and UBA966 according to GTDB-Tk. All genomes used in phylogeny were evaluated by CheckM to confirm completeness≥70%. The concatenated core gene alignments were also performed through UBCG and were selected using Gblocks. Model selecting and phylogenetic tree bulling were performed as before with the GTR + I + G4 model and 100 bootstrap replicates.

### 2.6. The Phylogenetic Tree of PVA Dehydrogenase

We used our nonredundant protein sequences of PVA dehydrogenase and all known protein sequences of PVA dehydrogenase (AMG75031.1, Q588Z1.3, and P77931.1) from NCBI to build the phylogenetic tree. Only sequences with length more than 500 bp were involved. Sequences were aligned using MAFFT [35] and were trimmed using trimAL [36]. The best-fit evolutionary model was selected using ModelTest-NG [33]. A multiple sequence alignment program, MAFFT, includes two novel techniques: the progressive method (FFT-NS-2) and the iterative refinement method (FFT-NS-i). The MAFFT program package is freely available at http://www.biophys.kyoto-u.ac.jp/∼katoh/programs/align/mafft. trimAl, a tool for automated alignment trimming in large-scale phylogenetic analyses, is freely available for download (http://trimal.cgenomics.org) and can be used online through the Phylemon web server (http://phylemon2.bioinfo.cipf.es/). ModelTest-NG is a reimplementation from scratch of jModelTest and ProtTest, two popular tools for selecting the best-fit nucleotide and amino acid substitution models, respectively. ModelTest-NG is available under a GNU GPL3 license at https://github.com/ddarriba/modeltest. The phylogenetic tree was inferred using RAxML-NG [34] with the LG + G4 model. RAxML-NG is a from-scratch reimplementation of the established greedy tree search algorithm of RAxML/ExaML. RAxML-NG offers improved accuracy, flexibility, speed, scalability, and usability compared with RAxML/ExaML. AxML-NG web service (maintained by Vital-IT) is available at https://raxml-ng.vital-it.ch/.Node support was generated through 100 bootstrap replicates. The phylogenetic tree was finalized for publication using iTOL website [21].

## 3. Results

We obtained shotgun metagenome sequence from four *Taisui* samples (located in Liaoning, Inner Mongolia, and Xinjiang province, Figure 1(a)). The metagenomic database provided 27.3 Gb clean data and 178 million high-quality reads in total for de novo assembling and binning (Table 1).

### 3.1. Taxonomic Annotation

The taxonomic annotation indicates the stabilization of four *Taisui* microbial communities. Proteobacteria was the dominant phylum with relative abundances from 59.55% to 71.82%. Five phyla, Planctomycetes, Acidobacteria, Chloroflexi, Actinobacteria, and Bacteroidetes, were subdominant populations (with abundances from 1% to 10%). The stabilization of *Taisui* communities was also found at other taxonomic levels. At the family level, most taxa (>80%) were common in all samples (Figure 1(c)). Twelve families—containing Caulobacteraceae, Sphingomonadaceae, Bradyrhizobiaceae, etc.—were enriched in samples with more than 1% relative abundance in at least one sample (Figure 1(b)). However, diversities emerged in family distribution. For example, TS.JZ1 had more than 2 fold abundance of Bradyrhizobiaceae compared with other samples; TS.BT and TS.XJ had more than 2 fold abundance of Sinobacteraceae compared with samples from Liaoning (Figure 1(b)).

*Taisui* from the same location (TS.JZ1 and TS.JZ2) had similar microbial composition. Simpson index in TS.JZ1 was the same as TS.JZ2, while Simpson index in TS.BT was the same as TS.XJ. Shannon index shows more diversity among samples, but indicates the same trend as Simpson index (Figure 1(d)). Besides, the UPGMA tree based on beta diversity illustrates TS.JZ1 and TS.JZ2 as one clade (Figure 1(d)).

### 3.2. Metagenome-Assembled Genomes

#### 3.2.1. Assembly of 97 Draft Genomes

We generated 97 metagenome-assembled genomes (MAGs) with completeness ≥70% and contamination ≤5%. According to Bowers et al. [37], 65 MAGs were high-quality drafts. Among them, 43 bins were preferable with >95% completeness and <5% contamination, and 2 bins were almost complete with >97% completeness and 0% contamination. All MAGs had at least 6× average coverage depth, and 6 Proteobacteria MAGs had more than 100x coverage (Figure 2). Our MAGs were taxonomically assigned to 13 microbial phyla by GTDB-Tk (Figure 2). Notably, 2 MAGs belonged to the bacteria candidate phylum.

We obtained 95 putative novel species (ANI between MAG vs. reference genome < 95% and 67 MAGs without closest placement ANI), and 97 putative novel strains (ANI < 99%), according to the standard suggested by Glendinning et al. [29]. Besides, metagenomic databases provided 39 putative novel genera from 43 MAGs (MAGs which clustered at 60% mean AAI (amino acid identity) did not have a genus assignment by GTDB-Tk [30]). Putative novel genera belonged to 8 phyla involving Proteobacteria, Planctomycetes, Chloroflexi, Acidobacteria, Bacteroidota, Bdellovibrionota, Gemmatimonadota, and Verrucomicrobiota.

#### 3.2.2. Novel Genus-Level Lineages

Two novel genus-level lineages were found in *Taisui* database, based on the standards: (1) they formed monophyletic lineages in the phylogeny, and (2) the average AAI was 60-80% between the genomes of such lineages and was <55% compared with known genera [30, 38].

In the tree of Planctomycetes members, we defined one genus-level novel lineage within the Planctomycetia class (Figure 3(a)). This lineage involved TS_28 (average coverage depth 24×) and Planctomycetales bacterium (GCF_009177095), with 66.4% AAI between members of it. The lineage—containing TS_28, GCF_009177095, TS_23 (7x), TS_47 (7x), and TS_60 (9x)—was a novel lineage at a higher taxonomic rank, because AAI between members ranged from 54.9% to 59.8%. Besides, the TS_84 (64x) may belong to a candidate novel class of Planctomycetes, which has shown AAI < 45% with other members of the Planctomycetes tree.

In the tree of Chloroflexi members, we defined one genus-level novel lineage within the Dehalococcoidia class (Figure 3(b)). It contained TS_80 (10x), TS_54 (13x), TS_90 (17x), and Dehalococcoidia bacterium UBA2991. The UBA2991 was identified in saline water as the unclassified Dehalococcoidia bacterium [39]. Members of this lineage show <49% AAI with genomes of Dehalococcoidales order and Dehalogenimonas order, which suggests this lineage was at least genus-level [30].

#### 3.2.3. Novel Gene Clusters for Secondary Metabolite Biosynthesis

Among our MAGs, 503 biosynthetic gene clusters (BGCs) were identified from 12 microbial phyla (Figure 4(a)). Our BGCs included 22 kinds of types, containing polyketide synthases (PKSs), nonribosomal peptide synthases (NRPSs), synthases of linear azole-containing peptides (LAP), etc. Proteobacteria are linked with most types of BGCs (*n* = 18), followed by Planctomycetes (*n* = 12), Chloroflexi (*n* = 10), and Acidobacteria (*n* = 10).

MAGs provided BGCs that relate to new drug development. We identified 167 PKS (types I and III), NRPS, NRPS-like, and NRPS-PKS gene clusters from 8 phyla. Searching against the MIBiG database, 149 NRPS, NRPS-like, and PKS gene clusters had the potential structural divergence of their products with known biosynthetic genes, because these BGCs showed <60% similarity with known clusters [40].

In the Chloroflexi phylum, *Candidatus Promineofilum* sp. TS_38 had unusually large repertoires of NRPS (include NRPS-like clusters) or PKS regions. TS_38 contained 14 targeted biosynthetic loci (754.9 kbp in total length) in 7.3 Mbp contigs. The largest interested region was 108.2 kbp. Seven regions were complex NRPS-type I PKS systems (involving hybrid, neighboring, or interleaved) in TS_38 (Figure 4(b)).

In the Planctomycetes phylum, MAGs of novel lineage—including TS_28, TS_23, TS_47, and TS_60—were identified with PKS or NRPS loci. The phylogenetic tree reveals that the NRPS-like and T3PKS gene clusters were commonly observed in the closest reference genomes, but the NRPS and T1PKS gene clusters were only observed in the *Taisui* MAGs (Figure 4(c)).

### 3.3. PVA Degradation

#### 3.3.1. Novel Putative PVA Dehydrogenase Genes

*Taisui* metagenomic database provided 264 putative PVA dehydrogenase gene based on the KEGG database. Most of PVA dehydrogenase genes were derived from Proteobacteria (208), followed by Acidobacteria (29) and Actinobacteria (21). To understand the evolution of the PVA dehydrogenase genes, we built the phylogenetic tree using protein sequences of our putative genes (length > 500 bp) and all 3 PVA dehydrogenase sequences from NCBI. The phylogenetic tree shows that PVA dehydrogenase may have been ancestral in Proteobacteria, Acidobacteria, and Actinobacteria phyla (Figure 5). PVA dehydrogenase in Deltaproteobacteria members (including Deltaproteobacteria bacterium and *Phenylobacterium* sp.) may be gained via horizontal gene transfer from members of Actinobacteria. One species of Planctomycetes had PVA dehydrogenase, which was placed between clades of Actinobacteria.

#### 3.3.2. Putative Pyrroloquinoline-Quinone Synthase Genes

In PVA degradation, pyrroloquinoline quinone (PQQ) is presumed to be needed for PVA dehydrogenase [2]. To identify microbial symbiotic during PVA degradation, we assigned putative PQQ synthase genes to taxon. More than half of PQQ synthase genes were derived from Proteobacteria. *Bradyrhizobium icene* provided most amount of PQQ synthase (387), followed by *Chlorobi bacterium* OLB5 (164) and *Novosphingobium nitrogenifigens* (137). The result shows the difference of providers for PVA dehydrogenase and PQQ synthase in *Taisui* systems.

## 4. Discussion

### 4.1. The Relative Stable Microbial System in *Taisui*

In the present work, we gave the first standard of *Taisui* metagenome through shotgun sequencing of four samples. According to the analysis of 228 *Taisui* finding-reports, *Taisui* mainly exists in the soil layer of northern China [4]. Therefore, we chose four soil existed *Taisui* samples from northern China with stable morphology for better representation (microscopic observations in Figure S1). The taxonomic analysis illustrates a relatively consistent microbial community structure in different *Taisui* samples. *Taisui* samples from the same location had closer community structures. Biogeographic patterns of bacteria had been identified in soil metagenomes, which are more related to environmental variation [41]. The taxonomic variation between *Taisui* samples may also be influenced by environmental variations, for example, precipitation (TS.JZ1 and TS.JZ2 were from subhumid regions; TS.BT was from the semiarid region; TS.XJ was from the arid region). Besides, dominant taxa in *Taisui* were common taxa in soil metagenomes. Marker gene amplification of *Taisui* also illustrates the same phenomenon [3]. It is reasonable because we used soil existed *Taisui*.

The functional annotation shows almost the same relative abundances of functional classifications of *Taisui* samples (Figure S2 and S3). The functional stability was also identified in human gut microbiota, which indicates the existence of a relatively stable ecological system [42]. Reconstruction of meta-pathway illustrated *Taisui* communities as carbon fixation, nitrogen fixation, and biosynthesis (Figure 6). At the family level, Caulobacteraceae, Sinobacteraceae, and Sphingomonadaceae contributed more than 30% related genes of the reductive citric acid cycle (rTCA cycle), while Burkholderiales, Xanthobacteraceae, Sphingomonadaceae, and Bradyrhizobiaceae contributed almost half of the N-fixation enzymes on average. The difference between functional providers of carbon fixation and nitrogen fixation may suggest the symbiosis between microbes in the *Taisui* community. However, more samples are needed for reliable cooccurrence network analysis [43].

### 4.2. Expanded Diversity of Microbial Genome and Biosynthetic Gene Cluster

Historical changes in population size, such as those caused by demographic range expansions, can produce nonadaptive changes in genomic diversity through mechanisms such as gene surfing Microbial species and their populations exhibit remarkable genomic diversity [44]. While mutation and recombination promote genetic variation in all forms of life, the genomic diversity of Bacteria and Archaea is enhanced dramatically by their proclivity for Horizontal Gene Transfer (HGT). Genomic analyses of diverse microbes provide similar results and it seems that a majority of genes in any pan-genome will be comprised of either high-frequency core genes or low-frequency strain-specific genes. These patterns of genomic diversity reveal the fundamental impact of HGT on evolution, and they suggest that bacterial and archaeal genomes comprise a dynamic mosaic of horizontally acquired genes whose frequency fluctuates in the population in response to both selection and genetic drift.

Our MAGs filled in some phylogenetic gaps and could be valuable in the detail inferring of phylogenetic relationships in bacterial. The MAGs for novel genera include taxa with very little genomic information published. One novel genus belonging to Proteobacteria was assigned to the Steroidobacteraceae family, and this family has only 9 published genomes in NCBI. In the Chloroflexi phylum, we identified one novel genus in each of the classes Dehalococcoidia and Aredenticatenia. The Dehalococcoidia contain only 2 formally published genera, involving Dehalococcoides and Dehalogenimonas [45]. And the Aredenticatenia class only had been identified in sludge and hydrothermal field [46–49] with 8 published genome on NCBI. In the Acidobacteria phylum, 3 novel genera of the Holophagales order were identified. The Holophagales order only contains the genera *Holophaga* and *Geotes* with a wide range of uncultured bacteria mainly from marine and soil [50].

Our MAGs also included novel gene clusters of NRPS, NRPS-like, and PKS (89.2% gene clusters < 60% similarity with known BGCs). Most of identified BGCs were linked with Proteobacteria, which is a common producer of wide bacterial natural products [51–53]. But few BGCs were reported in the published genomes of bacteria candidate phyla [54, 55]. We expand the number of taxa in Candidatus Dadabacteria phylum encoding BGCs. Besides, 2 MAGs of the Ardenticatenaceae family (belonging to Chloroflexi phylum) were detected with large NRPS or PKS loci, which were referred to as “*Candidatus Promineofilum* sp. TS_6” and “*Candidatus Promineofilum* sp. TS_38.” The BGCs linked to Ardenticatenaceae were few (6 linked clusters in total), according to the IMG database [54]. We expand Ardenticatenaceae with potential productions of PKS and NRPS. The large NRPS and PKS loci may provide source for new drug finding.

According to the phylogenetic tree of Planctomycetes members, NRPS and T1PKS were only observed in *Taisui* MAGs (novel lineage including TS_23, TS_47, TS_60, and TS_28). This result suggests that these two types of BGCs were acquired independently in evolutionary time in these taxa. The products of BGCs were used for the competition or communication with the producers' environment, and the abundance of NRPS and PKS domains was influenced by environmental conditions, involving soil depth, latitude, moisture, etc. [55, 56]. Therefore, the unconventional environment offered by *Taisui* may cause the encoding of NRPS and T1PKS gene clusters in these MAGs.

### 4.3. Rich Diversity of PVA Dehydrogenase Genes in the *Taisui* Microbial Community

PVA degradation includes two steps: first, the conversion from the 1,3-glycol structure of two successive repeating units to the beta-diketone; second, the broken of the carbon-carbon bond and the conversion of ketone group to carboxylic group [57]. In *Taisui* systems, the first step may begin with PQQ and PVA dehydrogenase, according to the functional annotation. *Taisui* has high water content, so the carbon-carbon bond may be cleavage by oxidized PVA hydrolase with H_2_O participation, like the model illustrated in methylotrophic yeast [58].

Microbes with PVA degradation ability are rare. Most PVA-degraders belong to the Pseudomonas and Sphingomonas genera. Although with novel degraders identified from grapes and marine bacterium [2], the taxonomic survey of PVA-degraders is not fruitful. Our results of putative PVA-degraders from 4 phyla can be a markable expansion for PVA biodegradation. Genera involving *Phenylobacterium*, *Conexibacter*, *Steroidobacter*, *Brevundimonas*, *Eilatimonas*, *Sphingopyxis*, and *Acidobacterium* may also be the source of PVA-degraders.

For PQQ-dependent PVA dehydrogenase, PVA degradation begins with the action of PQQ [2]. The production of PQQ by microbes (involving *Bradyrhizobium*, *Novosphingobium*, *Rhodopseudomonas*, etc.) can enhance the rate of PVA degradation. Besides, PVA dehydrogenase and PQQ synthase were abundant in different species, which suggests the microbial dependency on PVA degradation in *Taisui*.

## 5. Conclusion

According to metagenomic analysis, we concluded that the community structure of polymeric compound *Taisui* was relatively stable. The high abundances of Proteobacteria, Acidobacteria, Chloroflexi, Actinobacteria, and Bacteroidetes in *Taisui* can also be identified in the soil microbial community, suggesting the close relationship of *Taisui* and soil. As a unexplored system, *Taisui* communities provide genomes of previously poorly sampled microbial lineages, which is a valuable step for a comprehensive picture of the evolutionary history of life. For new drug development, BGCs of PKS and NRPS were expanded in phyla including Candidatus Dadabacteria, Chloroflexi, and Planctomycetes. The substantial putative PVA dehydrogenase genes were identified in 4 phyla, suggesting rich diversity of PVA dehydrogenase genes in *Taisui* communities. The gene of PVA degradation in microbes may acquire independently or from horizontal gene transfer. And the PQQ providers may enhance the PVA degradation rate in *Taisui*.

## Figures and Tables

**Figure 1:** Taxonomic analysis of Taisui metagenome: (a) sample locations in northern China, (b) the relative abundance (%) of major families in Taisui samples, (c) the upset plot of the family count in each sample, and (d) alpha and beta diversities of Taisui metagenomes (the UPGMA clustering based on Bray-Curtis distances of species richness).

**Figure 2:** The maximum-likelihood tree among genomes recovered from Taisui samples. The MAGs were labelled by phylum and class, as assigned by GTDB-Tk. MAGs with “undefined” label were only able to be defined at phylum level. Branches with bootstrap that support more than 50% were denoted with a purple circle, which became larger as the bootstrap support value increases. The average coverage depth of all contigs in a bin was shown as heat map.

**Figure 3:** Placement of the Planctomycetes (a) and Chloroflexi (b) MAGs into their phylogenetic context. The trees included MAGs and published genomes with the completeness ≥ 70% and were inferred using RAxML-NG with 100 bootstrap replicates. Only branches with bootstrap support values ≥50% were shown. The MAGs were labelled at the class level. Genus-level novel branches were shown in red. Novel branches at higher level than genus were shown in purple.

**Figure 4:** Predicted biosynthetic gene clusters from the Taisui MAGs: (a) biosynthetic gene clusters (BGCs) identified on MAG sequences were summed as phyla on the y axis and were colored by product types as the results of antiSMASH, (b) seven large PKS-NRPS hybrid or neighboring or interleaved gene clusters in the Candidatus Promineofilum sp. TS_38 genome were shown, and (c) phylogenetic tree of Planctomycetia MAGs with predicted PKS or NRPS clusters (∗) and closest reference genomes of them (counts of PKS or NRPS clusters was shown in the bar plot).

**Figure 5:** The maximum-likelihood tree of protein sequences of PVA dehydrogenase. Sequences from NCBI were shown in gray.

**Figure 6:** The sketch map of the metabolic pathways reconstructed from genes of Taisui samples (based on Figure S4–S7). The pie charts, which beside the names of enzymes or pathways, show the contribution ratio of taxa at family level. Abbreviations: NRT: ammonium transporter; NifDKH: nitrogenase; metB: cystathionine gamma-synthase; metE: 5-methyltetrahydropteroyltriglutamate--homocysteine methyltransferase; metH: 5-methyltetrahydrofolate--homocysteine methyltransferase; metK: S-adenosylmethionine synthetase; SepD: S-adenosylmethionine decarboxylase; SepA: arginine decarboxylase; SepB: agmatinase; SepE: spermidine synthase; PorABDG: pyruvate ferredoxin oxidoreductase; SAM: S-Adenosylmethionine; CysPUWA: sulfate transporters; ABC transporters: ATP-binding cassette transporters; MEP: 2-C-methyl-D-erythritol-4-phosphate.

**Table 1:** Summary of shotgun sequencing and assembly statistics.

	TS.JZ1	TS.JZ2	TS.BT	TS.XJ
Clean data size (Gb)	6.4	6.7	7.1	7.1
Clean_Q20	98.66	97.48	97.09	97.52
Clean_Q30	96.55	93.37	92.36	93.41
Number of high quality paired-end reads	45,183,937	43,169,867	44,363,607	45,284,710
Total number of bases	6,777,590,550	6,475,480,050	6,654,541,050	6,792,706,500
Number of contigs (≥500 bp)	391,852	533,634	419,397	479,713
Total contig length (bp)	472,635,294	637,814,029	686,512,143	702,537,509
Average contig size (bp)	1206	1195	1637	1464
Contig N50 (bp)	1339	1287	2465	1910
Largest contig size (bp)	290,257	1,977,463	851,561	1,021,402
Number of transcripts (Prokka)	711,761	820,620	776,716	824,658
Average transcripts length (bp)	473	514	624	585

## Data Availability

Sequences in this paper have been submitted to NCBI with SRA accession numbers SRR8569139-SRR8569142.

## Supplementary Materials

Supplementary Materials Figure S1: microscopic observations of *Taisui* tissues. (a) The histological imprints of a piece of *Taisui* tissue. (b) The histological sections stained with hematoxylin and eosin (HE) of *Taisui* tissues. Figure S2: the relative abundance (%) of KEGG based annotations in *Taisui* samples. The relative abundances of the level 1 classification of KEGG in four samples. (b) The relative abundances of the level 2 classification of KEGG in four samples (classifications with relative abundance above 1% are shown). Figure S3: the relative abundance (%) of COG-based annotations in *Taisui* samples. The relative abundances of the level 1 classification of COG in four samples. (b) The relative abundances of the level 2 classification of COG in four samples. Figure S4: the enrichment of carbon fixation pathways in four *Taisui* samples. Each node was divided into four blocks vertically, representing TS.JZ1, TS.JZ2, TS.BT, and TS.XJ in order from left to right. The colors of blocks represent the count of transcripts that annotated to this function, and the red block represents the transcripts number ≥500. Figure S5: the enrichment of benzoate degradation pathways in four *Taisui* samples. Each node was divided into four blocks vertically, representing TS.JZ1, TS.JZ2, TS.BT, and TS.XJ in order from left to right. The colors of blocks represent the count of transcripts that annotated to this function, and the red block represents the transcripts number ≥500. Figure S6: the enrichment of nitrogen metabolism pathways in four *Taisui* samples. Each node was divided into four blocks vertically, representing TS.JZ1, TS.JZ2, TS.BT, and TS.XJ in order from left to right. The colors of blocks represent the count of transcripts that annotated to this function, and the red block represents the transcripts number ≥500. Figure S7: the enrichment of terpenoid backbone biosynthesis pathways in four *Taisui* samples. Each node was divided into four blocks vertically, representing TS.JZ1, TS.JZ2, TS.BT, and TS.XJ in order from left to right. The colors of blocks represent the count of transcripts that annotated to this function, and the red block represents the transcripts number ≥500.

## References

[1] Amann M., Minge O., Rieger B., Künkel A., Coates G. W., Reichardt R., Dinjus E., Zevaco T. A. (2011). Biodegradability of poly(vinyl acetate) and related polymers. *Synthetic Biodegradable Polymers, Advances in Polymer Science*.

[2] Halima N. B. (2016). Poly(vinyl alcohol): review of its promising applications and insights into biodegradation. *RSC Advances*.

[3] Li E., Ren J., Chen Q. (2020). Uncovering the mysterious identity of Taisui—an old Chinese folk legend. *Science China. Life Sciences*.

[4] Wang C., Wang S. (2015). A research of the finding and distribution law of Taisui in modern China. *Agricultural Sciences*.

[5] Albertsen M., Hugenholtz P., Skarshewski A., Nielsen K. L., Tyson G. W., Nielsen P. H. (2013). Genome sequences of rare, uncultured bacteria obtained by differential coverage binning of multiple metagenomes. *Nature Biotechnology*.

[6] Chen L.-X., Anantharaman K., Shaiber A., Eren A. M., Banfield J. F. (2020). Accurate and complete genomes from metagenomes. *Genome Research*.

[7] Green M. R., Sambrook J. (2017). Isolation of high-molecular-weight DNA using organic solvents. *Cold Spring Harbor Protocols*.

[8] Patel R. K., Jain M. (2012). NGS QC toolkit: a toolkit for quality control of next generation sequencing data. *PLoS One*.

[9] Ewels P., Magnusson M., Lundin S., Käller M. (2016). MultiQC: summarize analysis results for multiple tools and samples in a single report. *Bioinformatics*.

[10] Li D., Liu C.-M., Luo R., Sadakane K., Lam T.-W. (2015). MEGAHIT: an ultra-fast single-node solution for large and complex metagenomics assembly via succinct de Bruijn graph. *Bioinformatics*.

[11] Gurevich A., Saveliev V., Vyahhi N., Tesler G. (2013). QUAST: quality assessment tool for genome assemblies. *Bioinformatics*.

[12] Seemann T. (2014). Prokka: rapid prokaryotic genome annotation. *Bioinformatics*.

[13] Fu L., Niu B., Zhu Z., Wu S., Li W. (2012). CD-HIT: accelerated for clustering the next-generation sequencing data. *Bioinformatics*.

[14] Li W., Godzik A. (2006). Cd-hit: a fast program for clustering and comparing large sets of protein or nucleotide sequences. *Bioinformatics*.

[15] Patro R., Duggal G., Love M. I., Irizarry R. A., Kingsford C. (2017). Salmon provides fast and bias-aware quantification of transcript expression. *Nature Methods*.

[16] Buchfink B., Xie C., Huson D. H. (2015). Fast and sensitive protein alignment using DIAMOND. *Nature Methods*.

[17] Huson D. H., Beier S., Flade I. (2016). MEGAN community edition - interactive exploration and analysis of large-scale microbiome sequencing data. *PLoS Computational Biology*.

[18] Huerta-Cepas J., Szklarczyk D., Forslund K. (2016). eggNOG 4.5: a hierarchical orthology framework with improved functional annotations for eukaryotic, prokaryotic and viral sequences. *Nucleic Acids Research*.

[19] Cantarel B. L., Coutinho P. M., Rancurel C., Bernard T., Lombard V., Henrissat B. (2009). The carbohydrate-active enzymes database (CAZy): an expert resource for glycogenomics. *Nucleic Acids Research*.

[20] Huson D. H., Bryant D. (2006). Application of phylogenetic networks in evolutionary studies. *Molecular Biology and Evolution*.

[21] Letunic I., Bork P. (2016). Interactive tree of life (iTOL) v3: an online tool for the display and annotation of phylogenetic and other trees. *Nucleic Acids Research*.

[22] Luo W., Brouwer C. (2013). Pathview: an R/Bioconductor package for pathway-based data integration and visualization. *Bioinformatics*.

[23] Uritskiy G. V., DiRuggiero J., Taylor J. (2018). MetaWRAP—a flexible pipeline for genome-resolved metagenomic data analysis. *Microbiome*.

[24] Parks D. H., Imelfort M., Skennerton C. T., Hugenholtz P., Tyson G. W. (2015). CheckM: assessing the quality of microbial genomes recovered from isolates, single cells, and metagenomes. *Genome Research*.

[25] Chaumeil P.-A., Mussig A. J., Hugenholtz P., Parks D. H. (2019). GTDB-Tk: a toolkit to classify genomes with the genome taxonomy database. *Bioinformatics*.

[26] Parks D. (2016). CompareM. https://github.com/dparks1134/CompareM.

[27] Barco R. A., Garrity G. M., Scott J. J., Amend J. P., Nealson K. H., Emerson D. (2020). A genus definition forBacteriaandArchaeaBased on a standard genome relatedness index. *mBio*.

[28] Pritchard L., Glover R. H., Humphris S., Elphinstone J. G., Toth I. K. (2015). Genomics and taxonomy in diagnostics for food security: soft-rotting enterobacterial plant pathogens. *Analytical Methods*.

[29] Glendinning L., Stewart R. D., Pallen M. J., Watson K. A., Watson M. (2020). Assembly of hundreds of novel bacterial genomes from the chicken caecum. *Genome Biology*.

[30] Luo C., Rodriguez-R L. M., Konstantinidis K. T. (2014). MyTaxa: an advanced taxonomic classifier for genomic and metagenomic sequences. *Nucleic Acids Research*.

[31] Na S.-I., Kim Y. O., Yoon S.-H., Ha S., Baek I., Chun J. (2018). UBCG: up-to-date bacterial core gene set and pipeline for phylogenomic tree reconstruction. *Journal of Microbiology*.

[32] Castresana J. (2000). Selection of conserved blocks from multiple alignments for their use in phylogenetic analysis. *Molecular Biology and Evolution*.

[33] Darriba D., Posada D., Kozlov A. M., Stamatakis A., Morel B., Flouri T. (2020). ModelTest-NG: a new and scalable tool for the selection of DNA and protein evolutionary models. *Molecular Biology and Evolution*.

[34] Kozlov A. M., Darriba D., Flouri T., Morel B., Stamatakis A. (2019). RAxML-NG: a fast, scalable and user-friendly tool for maximum likelihood phylogenetic inference. *Bioinformatics*.

[35] Rozewicki J., Li S., Amada K. M., Standley D. M., Katoh K. (2019). MAFFT-DASH: integrated protein sequence and structural alignment. *Nucleic Acids Research*.

[36] Capella-Gutiérrez S., Silla-Martínez J. M., Gabaldón T. (2009). trimAl: a tool for automated alignment trimming in large-scale phylogenetic analyses. *Bioinformatics*.

[37] Bowers R. M., Kyrpides N. C., Stepanauskas R. (2017). Minimum information about a single amplified genome (MISAG) and a metagenome-assembled genome (MIMAG) of bacteria and archaea. *Nature Biotechnology*.

[38] Dudek N. K., Sun C. L., Burstein D. (2017). Novel microbial diversity and functional potential in the marine mammal oral microbiome. *Current Biology*.

[39] Parks D. H., Rinke C., Chuvochina M. (2017). Recovery of nearly 8,000 metagenome-assembled genomes substantially expands the tree of life. *Nature Microbiology*.

[40] Crits-Christoph A., Diamond S., Butterfield C. N., Thomas B. C., Banfield J. F. (2018). Novel soil bacteria possess diverse genes for secondary metabolite biosynthesis. *Nature*.

[41] Bay S. K., McGeoch M. A., Gillor O. (2020). Soil bacterial communities exhibit strong biogeographic patterns at fine taxonomic resolution. *Msystems*.

[42] The Human Microbiome Project Consortium (2012). Structure, function and diversity of the healthy human microbiome. *Nature*.

[43] Berry D., Widder S. (2014). Deciphering microbial interactions and detecting keystone species with co-occurrence networks. *Frontiers in Microbiology*.

[44] Choudoir M. J., Panke-Buisse K., Andam C. P., Buckley D. (2017). Genome surfing as driver of microbial genomic diversity. *Trends in microbiology*.

[45] Yang Y., Sanford R., Yan J. (2020). Roles of Organohalide-Respiring *Dehalococcoidia* in carbon cycling. *Msystems*.

[46] Hemp J., Ward L. M., Pace L. A., Fischer W. W. (2015). Draft genome sequence of Ardenticatena maritima 110S, a thermophilic nitrate- and iron-reducing member of the Chloroflexi class Ardenticatenia. *Genome Announcements*.

[47] Kawaichi S., Ito N., Kamikawa R., Sugawara T., Yoshida T., Sako Y. (2013). Ardenticatena maritima gen. nov., sp. nov., a ferric iron- and nitrate-reducing bacterium of the phylum ‘ Chloroflexi ’ isolated from an iron-rich coastal hydrothermal field, and description of Ardenticatenia classis nov. *International Journal of Systematic and Evolutionary Microbiology*.

[48] Ward L. M., McGlynn S. E., Fischer W. W. (2018). Draft genome sequence of a divergent anaerobic member of the *Chloroflexi* class *Ardenticatenia* from a sulfidic hot spring. *Genome Announcements*.

[49] Zhang M., Yao J., Wang X., Hong Y., Chen Y. (2019). The microbial community in filamentous bulking sludge with the ultra-low sludge loading and long sludge retention time in oxidation ditch. *Scientific Reports*.

[50] Fukunaga Y., Kurahashi M., Yanagi K., Yokota A., Harayama S. (2008). Acanthopleuribacter pedis gen. nov., sp. nov., a marine bacterium isolated from a chiton, and description of Acanthopleuribacteraceae fam. nov., Acanthopleuribacterales ord. nov., Holophagaceae fam. nov., Holophagales ord. nov. and Holophagae classis nov. in the phylum 'Acidobacteria'. *International Journal of Systematic and Evolutionary Microbiology*.

[51] Brotherton C. A., Medema M. H., Greenberg E. P. (2018). *luxR* Homolog-Linked biosynthetic gene clusters in *Proteobacteria*. *MSystems*.

[52] Buijs Y., Bech P. K., Vazquez-Albacete D. (2019). Marine Proteobacteria as a source of natural products: advances in molecular tools and strategies. *Natural Product Reports*.

[53] Cimermancic P., Medema M. H., Claesen J. (2014). Insights into secondary metabolism from a global analysis of prokaryotic biosynthetic gene clusters. *Cell*.

[54] Palaniappan K., Chen I.-M. A., Chu K. (2020). IMG-ABC v.5.0: an update to the IMG/Atlas of Biosynthetic Gene Clusters Knowledgebase. *Nucleic Acids Research*.

[55] Sharrar A. M., Crits-Christoph A., Méheust R., Diamond S., Starr E. P., Banfield J. F. (2020). Bacterial secondary metabolite biosynthetic potential in soil varies with phylum, depth, and vegetation type. *mBio*.

[56] Charlop-Powers Z., Owen J. G., Reddy B. V. B., Ternei M. A., Brady S. F. (2014). Chemical-biogeographic survey of secondary metabolism in soil. *Proceedings of the National Academy of Sciences*.

[57] Leja K., Lewandowicz G. (2010). Polymer biodegradation and biodegradable polymers - a review. *Polish Journal of Environmental Studies*.

[58] Jia D., Li J., Liu L. (2013). High-level expression, purification, and enzymatic characterization of truncated poly(vinyl alcohol) dehydrogenase in methylotrophic yeast Pichia pastoris. *Applied Microbiology and Biotechnology*.

